# Detection of *Helicobacter* spp. DNA in the colonic biopsies of stray dogs: molecular and histopathological investigations

**DOI:** 10.1186/1746-1596-9-50

**Published:** 2014-03-06

**Authors:** Fatemeh Soghra Abdi, Shahram Jamshidi, Farhad Moosakhani, Farhang Sasani

**Affiliations:** 1 Department of Small Animal Internal Medicine, Resident of Specialized Veterinary Sciences, Science and Research Branch, Islamic Azad University (IAU), NO.14, Corner of Parvaz 1, Payam Blvd., Saadat Abad, Tehran, Iran; 2 Department of Clinical Sciences, Faculty of Veterinary Medicine, University of Tehran, Tehran, Iran; 3 Department of Microbiology, Faculty of Veterinary Medicine, University of Karaj, Karaj, Iran; 4 Department of Pathology, Faculty of Veterinary Medicine, University of Tehran, Tehran, Iran

**Keywords:** Dog, Inflammatory lesions, *Helicobacter*, Single PCR, Colonic biopsies

## Abstract

**Abstract:**

**Background**

In dogs, the gastric *Helicobacter* spp. have been well studied, but there is little information regarding the other parts of the alimentary system. The incidence of *Helicobacter* spp. infection in dogs is largely unknown and to our knowledge there are no data about their potential pathogenic role. In light of these considerations, the aims of this study were (i) to assess the prevalence of *Helicobacter* spp. in colonic biopsies of healthy and symptomatic stray dogs also (ii) we isolate and characterize helicobacters in canine colonic biopsies to compare the commonly used tests for the identification of *Helicobacter* spp. and to determine the occurrence of these species in dogs.

**Methods**

Tissues from fifteen stray dogs (8 males and 7 females, age 6 months –10 years) were used in this study. From each stray dog, multiple colonic biopsies were taken for PCR. Biopsies for PCR of cecum and colon were immediately frozen and stored at -20°C until DNA extraction. Samples for histological examination were fixed in 10% neutral buffered formalin and embedded in paraffin wax.

**Results**

In the cecum and colon, *Helicobacter* spp. DNA was detected in all dogs. *H.canis*, *H.bizzozeronii*, *H. bilis*, *H.felis*, *H.salomonis* and *H.pylori* Identified by specific polymerase chain reaction. Histopathology demonstrated that *Helicobacter* organisms were localized within the surface mucus and the intestinal crypts. Dogs with heavy *Helicobacter* spp. colonization were significantly in younger as well as had a higher level of mucosal fibrosis/atrophy than dogs with uncolonized or poorly colonized biopsies (*p* < 0.05).

**Conclusions**

We have indicated that the crypts of the cecum and colon of healthy and symptomatic dogs are heavily colonized by *Helicobacter* spp.. Combined molecular and histological approaches demonstrated that enterohepatic *Helicobacter* spp. infection is rather common in colonic biopsies of healthy and symptomatic stray dogs, with *Helicobacter* spp. specialy *H. canis*, *H.bizzozeroni*, *H.billis, H.felis* and *H. salomonis* identified as the most common species.

**Virtual Slides:**

The virtual slide(s) for this article can be found here: http://www.diagnosticpathology.diagnomx.eu/vs/1957989294118782.

## Background

Based on their preferential site of colonization and phylogenetic analysis of 16S and 23S rRNA genes, members of the genus *Helicobacter* are divided into gastric and enterohepatic *Helicobacter* spp. [1,2]. *Helicobacter* spp. can be either part of the normal flora or associated with inflammatory and proliferative disorders of the alimentary tract in humans and animals [1]. A pathogenic role of the gastric and enterohepatic *Helicobacter* spp. in dogs has not yet been well elucidated. However, canine gastric and enterohepatic *Helicobacter* spp. have been identified in humans with gastrointestinal and systemic disorders [1], suggesting a potential zoonotic role, and warranting further investigations.

Since the first isolation of *Helicobacter pylori* from the stomach of humans by Warren and Marshall [3] several additional *Helicobacter* species have been identified in the gastrointestinal tract of various mammalian species and birds [1,4]. Similarlyto humans, gastric infection with *Helicobacter* spp. has been associated with variable degrees of gastritis in various animals, including dogs, cats, ferrets, pigs, monkeys and cheetahs [5], gastric adenocarcinoma in ferrets naturally infected by *H. mustelae*[5] and in Mongolian gerbils experimentally infected by *H. pylori*[6].

The discovery of *H. pylori* in humans [7] and its relationship to gastritis, peptic ulcer, and gastric neoplasia has increased interest in gastric bacteria. Research has focused on four specific areas: (i) prevalence of gastric bacteria in dogs and cats; (ii) investigation of these domestic animals as a source of zoonotic *Helicobacter* infection of humans [8,9]; (iii) clinical significance of gastric Helicobacters in dogs and cats; and (iv) development of animal models of human disease.

Recent reports indicate that in the canine stomachs three different culturable helicobacters can be present and they are regarded as different species: *H. felis*, *H.bizzozeronii* and *H.salomonis*[10,11].

Enterohepatic *Helicobacter* spp., including *H. bilis*, *H. canis*, *H. cinaedi* and other unclassified *Helicobacter* spp. have been recovered from the faeces of healthy and diarrhoeic dogs [1,12-14]. In healthy dogs, enterohepatic *Helicobacter* spp. were described to preferentially colonize the crypts of the cecum and colon [15]. However, despite the extensive literature on enterohepatic *Helicobacter* spp. infection associated with IBD in laboratory animals, the association between *Helicobacter* spp. infection and gastrointestinal inflammatory and proliferative disorders has not been established in dogs so far.

The goals of this study were to investigate the prevalence of *Helicobacter* spp. in colonic biopsies of pet dogs and its six different species in colonic biopsies of stray dogs, and to evaluate the effect of the *Helicobacter* spp. colonization status (heavily colonized, poorly colonized and uncolonized biopsies) on the presence of histological lesions and DNA sequencing.

## Methods

### Animal and samplings

Tissues from fifteen stray dogs (8 males and 7 females, age 6 month –10 years) were used in this study. Stray dogs were housed in the same research facility (Table 1). None of the animals had been treated with antibiotics within 4 weeks before examination. Endoscopy and biopsy sampling were performed as part of clinical investigation with the owners’ agreement. The study was approved by the Ethical Committee of of the Science and Research Branch, Islamic Azad University of Tehran. Tissue samples from the gastrointestinal tract of each dog were collected in a sterile manner, with care taken to avoid cross-contamination between different sites. From each stray dog multiple colonic biopsies were taken for PCR. After each sampling, the endoscope and the biopsy forceps were thoroughly cleaned, then sterilized using an activated aldehyde solution. Biopsies were immediately frozen and stored at -20°C until DNA extraction. Samples were fixed in 10% neutral buffered formalin and embedded in paraffin wax for histological examination.

**Table 1:** Age, gender, clinical signs, inflammatory and morphological changes and colonization status of Helicobacter spirochetes

**Dog no.**		**1**	**2**	**3**	**4**	**5**	**6**	**7**	**8**	**9**	**10**	**11**	**12**	**13**	**14**	**15**
Gender^a^		M	F	M	M	M	F	F	M	F	F	F	F	M	M	M
Age^b^		1	3	1	2	3	1	2	3	3	1	3	1	2	1	3
Clinical signs^c^		MD, W,A	H	MD, W,A	H	MD, W,A	MD, W,A	H	H	H	MD, W,A	H	H	MD, W,A	H	H
Persistence of Helicobacter spirochetes	Mucosal surface	+	+	+	+	+	+	+	+	+	+	+	+	+	+	+
	Crypt	+	+	+	-	-	+	-	-	-	+	-	+	+	-	-
Helicobacter spirochete colonization status^d^		+3	+2	+2	+1	+1	+2	+1	+1	+1	+3	+1	+2	+1	+2	+1
Inflammatory cell Infiltration^e^	LP	+	+	+	+	+	+	+	+	+	+	+	+	+	+	+
	N	+	+	+	-	-	+	-	-	-	+	-	+	+	-	-
	E	+	-	+	-	-	-	-	-	-	+	-	-	-	-	-
	M	-	+	+	-	-	+	+	-	+	+	-	-	+	+	+
Lymphoid follicles^f^		+2	+2	+2	0	0	+3	+1	0	+1	+3	0	+2	+1	+1	+1
Morphological changes	Surface epithelial injury	+	+	+	-	+	+	-	-	+	+	-	+	+	+	-
	Crypt hyperplasia	-	-	+	-	+	-	+	-	+	+	-	-	-	-	+
	Crypt dilation/distortion	+	-	+	-	+	-	+	-	+	+	-	-	-	-	-
	Mucosal fibrosis and atrophy	+	+	+	-	-	+	+	-	-	+	-	+	-	+	-
Severity of inflammatory and morphological changes^g^		Mi	Mo	Ma	No	Mi	Ma	Mi	No	Mi	Ma	No	Mo	Mi	Mo	Mi

^a^M = male; F = female.

^b^1 ≤ one year-old age; one year-old age < 2 ≤ five year-old age.

^c^A = anorexia; H = healthy; MD = mild diarrhea; W = weight loss.

^d^0 = [M = 0]; +1 = [M ≤ 10]; +2 = [10 < M ≤ 50]; +3 = [M ≥ 50]; [M = Mean Helicobacter spirochetes number in 10 microscopic field (Giemsa, ×1000)].

^e^LP = lymphocytes and plasma cells; N = neotrophils; E = eosinophils; Mmacrophage.

^f^0 = without lymphoid follicle; +1 = presence of one lymphoid follicle; +2 = presence of two lymphoid follicles; +3 = presence of three or more than three lymphoid follicles.

^g^No = normal (healthy dog); Mi = mild (Leukocytes appearance ≤ 10, with mild morphologic changes); Mo = moderate (10 < leukocytes ≤ 50, with moderate morphological changes); Ma = marked (leukocytes ≥ 50, with marked morphological changes).

### Polymerase chain reaction (PCR) amplification

DNA was extracted from biopsies by using a DNA easy tissue KIT® (Qiagen, Hilden, Germany) according to the manufacturer’s Instructions. The 16S rRNA gene of members of the family Helico-Bacteracea was amplified by primers H276f/H676r [16], by using a single PCR. Primers P17f/P17r [17] were used to amplify specifict protein of Helicobacter bilis. Primers Fe1F/Fe3R [18] were used to amplify urease gene of *H. bizzozeronii*. Furthermore, primers HSALF/ HSALR [19] were used to amplify HSP60 of *H.salomonis* and primers HP-for/HP-REV [20] were used to amplify the urease C gene of *H.pylori*. Primers canis3F/canis4R (EU233451) were used to amplify the HSp60 of *H.canis*. All PCR reactions were performed in an AIB Applied Biosystems Thermocycler (2720 thermal cycler, M/PCR/23), all the amplifications were performed in a final volume of 25 μl containing 5 μl of DNA extracted, 10.3 μl ultra-pure distilled water, 2.5 μl of 10×Tag polymerase buffer (Qiagen), 0.5 μl MgCl_2_ (Qiagen), 0.2 μl of Tag polymerase enzyme and 0.5 μl of each primer (MWG), 0.5 μl DNTP (Qiagen), 0.5 μl DNA Nucleotide (Qiagen), 5 μl Q Solution (Qiagen). Samples were heated at 94°C for 15 min and 30 s, denaturation phase, followed by 30 s at primer annealing temperatures that were different for the species and the family Helicobacteraceae. Primer annealing temperature for the family Helicobacteraceae was 52°C, for *H.bilis* was 55°C, for *H.felis* was 52°C, for *H.bizzozeronii* was 54°C, for *H. salomonis* was 51°C, for *H.pylori* was 49°C and for *H.canis* was 52°C, followed by 30 s in 72°C (extension phase) this cycle repeated 35 times, followed by 7 min in 72°C, final extension step and repair (Table 2). Ten microliters of each amplification product were analyzed by gel electrophoresis in 1.5% agarose gels in Tris-boric acid EDTA buffer (TBE).The gel was stained with ethidium bromide (0.5 mg/L) and examined under UV transilluminator for the presence of amplified DNA; the size of the expected fragments was compared to a 100 bp reference marker (Fermentas-e), (Table 3).

**Table 2:** Detection of Helicobacter spp., H.felis., H.canis., H.bizzozeronii., H.pylori., H.bilis and H.salomonis DNA in the biopsies of colon of fifteen healthy and symptomatic stray dogs by single PCR and sequencing

**Dog No.**	**1**	**2**	**3**	**4**	**5**	**6**	**7**	**8**	**9**	**10**	**11**	**12**	**13**	**14**	**15**
Helicobacteraceae (H276f/H676r)	+	+	+	+	+	+	+	+	+	+	+	+	+	+	+
H.bilis (P17f/P17r)	-	-	+	-	+	+	+	+	+	-	+	-	-	-	-
H.bizzozeronii (Bi1F/Bi2R)	+	+	+	+	+	+	+	+	+	+	+	+	+	+	+
H.canis (canis3F/canis4R)	+	+	+	+	+	+	+	+	+	+	+	+	+	+	+
H.felis (Fe1F/Fe3R)	-	-	+	-	-	+	-	+	+	-	+	-	-	-	+
H.pylori(HP-for/HP-REV)	-	-	-	-	-	-	-	-	-	-	+	-	-	-	+
H.salomonis(HSALS/HSALR)	+	+	+	-	+	+	+	-	+	-	+	+	+	+	+

-, negative; +, positive.

**Table 3:** Helicobacteraceae DNA was detected by nested PCR in colonic biopsies

**Primer**^**a**^	**Sequence (5' - 3')**^**b**^	**Product size (bp)**	**PCR conditions**	**Target sequence**	**References**^**c**^
H276f	CTA TGA CGG GTA TCC GGC	374	*94°c for 15 min and 30 s,52°c for 30 s,72°c for 30 s, 35 cycles,72°c for 7 min*	*Helicobacter* spp.16S rRNA	Riley et al. [17]
H676r	ATT CCA CCT ACC TCT CCC A				
p17f	ATG GAA CAG ATA AAG ATT TTA AAG CAA CTT CAG	435	*94°c for 15 min and 30 s,55°c for 30 s,72°c for 30 s, 35 cycles,72°c for 7 min*	*H. bilis* specifict protein	Feng et al. [21]
p17r	CTA TGC AAG TTG TGC GTT AAG CAT				
Fe1F	TTT GGT GCT CAC TAA CGC CCT C	434 (438)	*94°c for 15 min and 30 s,52°c for 30 s,72°c for 30 s, 35 cycles,72°c for 7 min*	*H. felis* urease gene	Baele et al. [19]
Fe3R	TTC AAT CTG ATC GCG TAA AG				
Bi1F	AAC CAA **Y**AG CCC CAG CAG CC	373	*94°c for 15 min and 30 s,54°c for 30 s,72°c for 30 s, 35 cycles,72°c for 7 min*	*H. bizzozeronii* urease gene	Baele et al. [19]
Bi2R	TGG TTT TAA GGT TCC AGC GC				
HSALF	CAT TTT CAA AGA GGG CTT GC	537	*94°c for 15 min and 30 s,51°c for 30 s,72°c for 30 s, 35 cycles,72°c for 7 min*	*H. salomonis* HSP60	Mikkonen et al. [20]
HSALR	GCA CAC CCC TCA GTT TGT TT				
HP-FOR	TTA TCG GTA AAG ACA CCA GAA A	132	*94°c for 15 min and 30 s,49°c for 30 s,72°c for 30 s, 35 cycles,72°c for 7 min*	*H. pylori* urease C gene	He et al. [22]
HP-REV	ATC ACA GCG CAT GTC TTC				
canis3F^d^	TAA GCG CGG TAT GGA TAA GG	254	*94°c for 15 min and 30 s,52°c for 30 s,72°c for 30 s, 35 cycles,72°c for 7 min*	*H. canis* HSP60	EU233451
canis4R^d^	TTA AGT AGC CGC GGT CAA AC				

^a^:Different Types of Primers, ^b^:Sequence of Helicobacteraceae DNA, ^c^:References studied for all the selected procedures, ^d^:comparison between numerical continuous of the primer in the helicobacter canis.

### DNA purification and sequencing

PCR products (there were 53 PCR products) were purified by Sanger method and then sequenced on the ABI 3730XL DNA Analyzer which provides high quality of sequence analysis data (Sequencing Service from Bioneer, Republic of Korea). Sequencing results were extracted and corrected in FASTA format by FinchTV as a trace file viewer. The identities of the gene sequences (16S rRNA gene, specific protein of H.bilis, urease gene of *H.felis*, urease gene of *H.bizzozeronii*, HSP60 of *H.salomonis*, urease C gene of *H pylori*, HSP60 of *H.canis*) were verified by comparison of the sequences to the GenBank database through the algorithm BLASTn. Finally, the verified sequences were aligned in the MEGA5 software [4] and the related phylogenetic tree was constructed for each group of sequences.

### Histological evaluation

Formalin-fixed paraffin-embedded 4 μm sections of colonic biopsies were stained with hematoxylin and eosin (H&E) and Periodic Acid-Silver Methenamine (PEM). The biopsies after staining were scored by a single phathologist. These criteria included the evaluation of inflammatory (infiltrates of lymphocytes and plasma cells, eosinophils, neutrophils and macrophages in the lamina propria) and morphological changes (surface epithelial injury, crypt hyperplasia, crypt dilation, distortion, mucosal fibrosis and atrophy). The degree of severity of both inflammatory and morphological changes was scored as follows: normal (0), mild (+), moderate (++) and marked (+++).

### Statistical analysis

The software, SPSS Version 16.0 for Windows (SPSS Inc., Chicago, IL), was used for analysis. To compare the data chi-square tests were used. Differences were considered significant when *P* < 0.05.

Mean spirochete colonization status in 10 microscopic fields (PEM,×1000) evaluated also scored for the presence of Helicobacter spirochetes in the superficial mucus and in the crypts as follows: 0 = uncolonized; +1 = colonization <10 organismes; +2 =10 organismes ≤ colonization <50 organismes; +3 = colonization ≥50 organismes.

## Results

### PCR

Results of the overall PCR amplification of *Helicobacter* spp. DNA, and the group-specific canine colonic *Helicobacter* spp. are summarized in Table 3. Helicobacteraceae DNA was detected with single PCR in all the colonic biopsies (100%), Futhermore, *H.canis* and *H.bizzozeronii* DNA in 100%, *H. bilis* DNA in 44%, *H.felis* DNA in 40%, *H.salomonis* DNA in 80% and *H.pylori* DNA in 1 of the 15 dogs examined (7%) were detected.

### DNA sequence analysis

Evolutionary relationships of taxa for *H. canis, H. bilis* and *H.Salomonis* were inferred using the UPGMA method [1]. The optimal tree with the sum of branch length = 1.04374900, 0.04752769, 0.74197122 are shown, respectively. The evolutionary distances were computed using the Kimura 2-parameter method [2] and are in the units of the number of base substitutions per site. The analysis involved 15 nucleotide sequences. Evolutionary analyses were conducted in MEGA5 [4] (Figures 1, 2, and 3).

**Figure 1:** **Helicobacteraceae DNA was detected with single PCR in all the colonic biopsies: Evolutionary relationships of taxa for *helicobacter canis *** **the evolutionary history was inferred using the UPGMA, Kimura 2-parameter and MEGA5 methods.**

**Figure 2:** **Helicobacteraceae DNA was detected with Single PCR in all the colonic biopsies: Evolutionary relationships of taxa for *helicobacter bilis *** **the evolutionary history was inferred using the UPGMA, Kimura 2-parameter and MEGA5 methods.**

**Figure 3:** **Helicobacteraceae DNA was detected with single PCR in all the colonic biopsies: Evolutionary relationships of taxa for *helicobacter salomonis *** **the evolutionary history was inferred using the UPGMA, Kimura 2-parameter and MEGA5 methods.**

PCR amplification of DNA from bacterial strains was counducted by (NO.1-7) *H.bilis* P17f/P17r primer; (NO. 8-22) *H.canis canis* 3F/canis4r primer; (NO.23-34) *H.salomonis* HSALF/HSALR primer; (NO.35-37) *H.felis* Fe1f/Fe3r primer; (NO.38-52) *H.bizzozeronii* Bi1F/Bi2R primer; (NO.53) *H.pylori* HP-for/HP-REV Primer, and 100-bp molecular ladder (Figure 4).

**Figure 4:** **The *Polymerase Chain Reaction *** **( *PCR *) on *DNA isolated *** **with standard *protocol*; PCR amplification of DNA from bacterial strains by (NO.1-7) H.bilis P17f/P17r primer; (NO. 8-22) *H.canis *** **canis3F/canis4r primer; (NO.23-34) *H.salomonis *** **HSALF/HSALR primer; (NO.35-37) H.felis Fe1f/Fe3r primer; (NO.38-52) *H.bizzozeronii *** **Bi1F/Bi2R primer; (NO.53) *H.pylori *** **HP-for/HP-REV Primer, and 100-bp molecular ladder.**

### Histological examination

Inflammatory changes in fiften cases there were various numbers of lymphocytes and plasma cells in the lamina propria of the colonic biopsies, occasionally admixed with lower numbers of neutrophils and rare eosinophils, whereas detectable aggregates of macrophages were found. Mild to severe lymphoplasmacytic and neutrophilic infiltration was found in colonic biopsies. (Figure 5A-D) Moreover, slides stained with Giemsa and Periodic Acid-Silver Methenamine (Figure 5A and B), the samples coinfected with less than 3 different species of Helicobacter (according to the PCR results) that had mild and unclear infection with helicobacter spirochetes. Although the mean value of neutrophilic infiltration was higher in heavily colonized biopsies compared to uncolonized and poorly colonized ones, this difference was not statistically significant.

**Figure 5:** **Colonic biopsies of *Helicobacter spp. *in the stray dogs. (A and B).** Colonic biopsies: Moderate to severe amount of *Helicobacter spp* in the superficial mucus entering a colonic crypt (Wright Giemsa staining) **C** and **D**: Lymphoplasmacytic and neutrophilic infiltration (hematoxylin and eosin; 400×).

### Morphological changes

Morphological changes of the colonic mucosa were present in 12/15 examined stray dogs with different degrees of severity. A statistically significant difference was found between heavily colonized colonic biopsies and both uncolonized and poorly colonized colonic biopsies for the parameter of mucosal fibrosis/atrophy (P < 0.05; Tables 1 and 2) as well as lieber kuhn’s glands secretion, crypt dilation, crypt hyperplasia and distortion were higher in samples with objective number of spirochetes than what there were in slides with poorly and non objective spirochetes, even though these differences were not statistically significant.

## Discussion

*Helicobacter* spp. are usually found in large numbers in the stomach of dogs but few data are available on the presence of these bacteria in other parts of the alimentary system. To date, enterohepatic *Helicobacter* spp. have been identified by culture in the feces of dogs and there are no data about their spatial distribution within the canine intestinal tract [13]. The fastidious nature of most *Helicobacter* spp. and the coexisting intestinal flora hinder their routine isolation from the intestine [23], therefore, we opted for a DNA sequence analysis approach to detect *Helicobacter* spp. in the canine alimentary tract. A combination of PCR, 16S rRNA gene cloning, sequencing and histopathology allowed us to identify specific regions of the alimentary tract that were colonized with *Helicobacter* spp. and to visualize morphologically intact microorganisms and their spatial distribution within the gastrointestinal tract of dogs, as previously reported in mice and children [24-26].

In present study a high prevalence of *Helicobacteraceae* (100%) with *H. canis* and *H. bizzozeronii* (100%) DNA was detected by PCR in examined colonic biopsies from healthy and symptomatic stray dogs. The incidence of other species including *H. salomonis* (80%), *H. bilis* (47%), *H.felis* (40%) and *H. pylori* (7%) were comparatively high to low, respectively. These results were in line with previous studies in which enterohepatic *Helicobacter* spp. were detected by PCR in 100% of the large intestines of a small group of healthy dogs [13]. Our study revealed higher outbreak of *helicobacter* spp. than some previous studies. Based on direct sequencing of the enterohepatic *Helicobacter* spp. PCR products, *H. salomonis*, *H. bilis*, *H.felis* and *H. pylori* were the most prevalent *Helicobacter* species present in the canine colonic biopsies that is in accordance with previous works [13,15].

The high incidence of enteric *H. canis* and *H. bizzozeronii* might be explained by anal–oral transmission due to typical canine social behaviour. The presence of *H. canis* and *H. bizzozeronii* in both cecum and colon is interesting from a zoonotic perspective since *H. canis* and *H. bizzozeronii* has caused infections in humans where contact with dogs was suspected [27]. *H. bizzozeronii* (100%) and *H.salomonis* (80%) were found in colon, supporting the idea that gastric *Helicobacter* spp. might transmit via oral contact [10,28]. The absence of gastric *Helicobacter* spp. in faecal samples is in agreement with previous studies [15].

Futhermore*, Helicobacter* spp. DNA was detected in the cecum and colon of all dogs. The degree of colonization assessed by histopathology showed variable amounts of positive bacteria in all the cecum and colon sections depending on the dog. In some of these samples, only a small amount of *Helicobacter* spp. DNA was detected by single PCR. The low level of colonization was reflected in the weak band obtained by the *Helicobacter* spp. PCR. *Helicobacter* spp. detected by PCR also histopathology had a comparable distribution and were localized either in the intestinal lumen at the mucosal surface admixed to other bacteria or within the intestinal crypts extending from the superficial to the deep portions of the crypts. This finding together with the occasional amplification of gastric *Helicobacter* spp. DNA and the absence of gastric *Helicobacter* spp. sequences in clone libraries likely reflects their relative scarcity in the large intestine compared to colonic *Helicobacter* spp. that suggests passive intestinal carriage of gastric *Helicobacter* spp. DNA.

In the present study, a significantly higher level of mucosal fibrosis/atrophy was found in heavily colonized colonic biopsies compared to uncolonized or poorly colonized ones. Fibrosis is considered a common consequence of IBD that results from the reaction of intestinal tissue to the damage induced by chronic inflammation but its pathogenesis has not been fully elucidated [29]. Since *Helicobacter* spp. have been considered as likely candidates for involvement in IBD pathogenesis [30-33] that fibrosis is a common IBD-associated lesion. The association between heavy *Helicobacter* spp. colonization and mucosal fibrosis/atrophy found in this study support the role of enterohepatic *Helicobacter* spp. in the development of canine IBD [1,16,30,31,34]. Therefore, our data may well explain the discrepancy previous studies.

## Conclusion

We have indicated that the crypts of the cecum and colon of healthy and symptomatic dogs are heavily colonized by *Helicobacter* spp.. Combined molecular and histological approaches demonstrated that *Helicobacter* spp. infection is rather common in colonic biopsies of healthy and symptomatic stray dogs, *Helicobacter* spp. Specialy *H. canis*, *H.bizzozeroni*, *H.billis, H.felis* and *H. salomonis* identified as the most common species. Additional studies are necessary to investigate if *Helicobacter* spp. are involved in cecal and colonic inflammatory or proliferative disorders in dogs, as demonstrated in other species.

## Competing interests

The authors declare that they have no competing interests.

## Authors’ contributions

FSA and FS participated in the histopathological evaluation, performed the literature review, acquired photomicrographs and drafted the manuscript and gave the final histopathological diagnosis. JJ performed sequencing alignment and manuscript writing. FSA, SHJ and FM edited the manuscript and made required changes. All authors have read and approved the final manuscript.
